# HMGA2 Promotes Brain Injury in Rats with Cerebral Infarction by Activating TLR4/NF-*κ*B Signaling Pathway

**DOI:** 10.1155/2022/1376959

**Published:** 2022-08-04

**Authors:** Shaoyue Huang, Zhen Hong, Leguo Zhang, Jian Guo, Yanhua Li, Kuo Li

**Affiliations:** No. 2 Department of Neurology, Cangzhou Central Hospital, Cangzhou, Hebei, China

## Abstract

Cerebral infarction is a common disease with a higher disability and fatality rates. The incidence rates of cerebral infarction or cerebral ischemic stroke gradually increase with aging and cerebrovascular disease progression. This study is aimed at evaluating the effects of HMGA2 on cerebral infarction-induced brain tissue damage and its underlying mechanisms. Adult Sprague Dawley rats were pretreated with sh-HMGA2 before cerebral infarction operation. The effect of HMGA2 on the arrangement, distribution, and morphological structure of neurons and the cell apoptosis ratio in brain tissue were detected via hematoxylin and eosin staining, brain-water content, TTC staining, and TUNEL staining. The results from ELISA assay, qPCR, and western blot indicated that downregulation of HMGA2 mitigated inflammatory stress via regulating the expression of TLR4/NF-*κ*B. In addition, results showed that suppressed HMGA2 attenuated the neurological dysfunction of brain injury rats and markedly reduced infarct volume. HMGA2 might be able to alleviate the damage associated with cerebral infarction-induced inflammatory response and cell apoptosis. Moreover, downregulation of HMGA2 had a protective effect on the brain damage derived from cerebral infarction by mediating the TLR4/NF-*κ*B pathway. In conclusion, the current study demonstrated that downregulation of HMGB2 decreased the infarct size, inflammatory responses, and apoptosis in cerebral injury and further had neuroprotective effects against cerebral infarction-induced brain damage. Finally, these results indicated that the downregulation of the TLR4/NF-*κ*B pathway after ischemia by HMGB2 inhibition is a potential mechanism of the neuroprotective effect of cerebral injury.

## 1. Introduction

Cerebral infarction, also known as ischemic stroke, is related to cerebral blood supply disorder, hypoxia, or ischemia in local brain tissue. Apoptosis is a hotspot in the research of cerebral ischemia-reperfusion injury in recent years [1], and it is a caspase-dependent cell death process. The cellular apoptosis involves numerous protein families, cytokines, and signaling pathways, including the BCL-2 protein family and caspase enzyme protein family, which ultimately activate receptor-dependent apoptotic pathways or endogenous apoptotic pathways [2, 3]. Toll-like receptor 4 (TLR4) is expressed in the immune system and can modulate the immune response. The lipopolysaccharide-induced phosphorylation of nuclear factor-*κ*B (NF-*κ*B) can trigger the TLR4 activation and further induce multiple cytokine production, transcription factors, and chemokine expression. Those factors play an essential role in the inflammatory response, immune system, cell survival, differentiation, and cellular apoptosis and further participate in the development of neuroinflammation [4, 5].

The TLR4/NF-*κ*B signaling pathway and the inflammatory response were activated in the cerebral infarction animal model. Previous studies have shown that aspirin reduced cerebral infarction by modulating the TLR4/NF-*κ*B-mediated endoplasmic reticulum stress in the mice model [6]. Recent research indicated that electroacupuncture promotes hippocampal neurogenesis and recovery of the nerve function through inhibiting the TLR4 signaling pathway after trauma and improves the formation of hippocampal neurons after traumatic brain injury in mice [7]. Therefore, the TLR4/NF-*κ*B signaling pathway is closely related to cerebral infarction-induced brain injury.

High-mobility group AT-hook2 (HMGA2) is a DNA binding protein. Under normal physiological conditions, HMGA2 is not expressed or rarely expressed in normal tissues. However, in diseases, as a structural transcription regulator, HMGA2 can play a critical role by regulation of related gene [8, 9]. HMGA2 is involved in the progression of brain diseases. Previous studies have revealed that HMGA2 significantly increases and promotes the release of proinflammatory cytokines (TNF-*α*, IL-6, and IL-1*β*) in brain tissue of mice with cerebral hemorrhage, and downregulating the expression of HMGA2 can suppress the inflammatory response and protect brain tissue from secondary brain damage after cerebral hemorrhage [10]. Previous studies have demonstrated that HMGA2 can enhance the activity of NF-*κ*B through binding to the AT-rich repeat sequence adjacent to the NF-*κ*B common site [11]. In addition, HMGA2 also promotes the LPS-induced proinflammatory cytokine release in RAW264.7 cells through activing the NF-*κ*B pathway [12].

However, there are few studies on the expression and function of HMGA2 in cerebral infarction as well as its related mechanisms. Therefore, this study explored the effect of HMGA2 on cerebral infarction-induced brain tissue damage and its underlying mechanisms.

## 2. Methods

### 2.1. Animal Model

Adult Sprague–Dawley rats weighing 220–260 g were purchased from Shanghai Experimental Animal Center of Chinese Academy of Sciences and housed under 12 hours light/12 hours dark cycle and had free access to diet and tap water all through the study. All animal experimental procedures were approved by the Cangzhou Central Hospital and were conducted in accordance with the US National Institutes of Health Guide for the Care and Use of Laboratory Animals. The animal model of MCAO operation was performed as described previously [13]. All rats were randomly divided into four groups, containing sham operated control group, transient middle cerebral artery occlusion for 90 min (MCAO), sh-HMGA2 injection with MCAO (sh-HMGA2 + MCAO), and sh-NC injection with MCAO (sh-NC + MCAO). Middle cerebral artery occlusion (MCAO) surgery was performed two weeks after sh-HMGA2 or sh-NC injection.

### 2.2. Quantitative Real-Time PCR (qRT-PCR)

The total RNA was isolated from brain tissues using the TRIzol method (Invitrogen, USA) according to the manufacturer's protocols. The cDNA synthesis was performed by the Prime-Script RT reagent kit (Tiangen, Beijing, China). qRT-PCR was conducted on an CFX96 Real-Time PCR Detection System (Bio-Rad, Hercules, CA, USA) and detected by using SYBR Green PCR Master Mix (TaKaRa).

The primers were as follows: HMGA2: forward: 5′-TCCCTCTAAAGCAGCTCAAAAGA-3′; reverse: 5′-TGTTGTGGCCATTTCCTAGGT-3′; TNF-*α*: forward: 5′-ATGAGCACTGAAAGCATGATCCGG-3′; reverse: 5′-GCAATGATCCCAAAGTAGACCTGCCC-3′; IL-6: forward: 5′-CCCACCAAGAACGATAGTCA-3′; reverse: 5′-CTCCGACTTGTGAAGTGGTA-3′; IL-1*β*: forward: 5′-ATGGCAGAAGTACCTAAGCTCGC-3′; reverse: 5′-ACACAAATTGCATGGTGAAGTCAGTT-3′; IL-18: forward: 5′-AGTAAGAGGACTGGCTGTGACCC-3′; reverse: 5′-TGTTATGGAAATACAGGCGAGGT-3′.

### 2.3. Western Blot

The cerebral tissue from each group was extracted and homogenized. 30 *μ*g protein form each sample was separated by 12% SDS-PAGE gel and then transferred to nitrocellulose membranes. After blocked with skimmed milk, the membranes were incubated with primary antibodies against Bax (1 : 2000, Santa Cruz Biotechnology, USA), cleaved caspase-3 (1 : 3000, Abcam, Cambridge, UK), Bcl-2 (1 : 5000, Abcam, Cambridge, UK), TLR4 (1 : 5000, Abcam, Cambridge, UK), p-p65 (1 : 2000, Abcam, Cambridge, UK), p65 (1 : 5000, Abcam, USA), p-I*κ*B (1 : 3000, Sigma-Aldrich, USA), I*κ*B (1 : 3000, Sigma-Aldrich, USA), and GAPDH (1 : 20000, Santa Cruz Biotechnology, UK) overnight at 4°C and subsequently incubated with secondary antibody for 1 hour. The specific protein signals were detected by enhanced chemiluminescence reagent (Bio-Rad, USA). The density of western blots was measured using ImageJ.

### 2.4. TTC Staining

After experiment, animals were sacrificed, and their brains were placed on ice and cut into three coronal slices with 2 mm thick sections. Then, the brain sections were stained for 20 minutes with 2% 2,3,5-triphenyltetrazolium chloride solution at 37°C. The infarcted tissues stained white, whereas the normal brain was red. Infarct volume was quantified by ImageJ software.

### 2.5. H&E Staining

After MCAO, the rats were sacrificed, and brain tissues were fixed with 4% formaldehyde. The fixed brain tissues were dehydrated with different concentration gradients alcohol and cut into 5 mm sections. The tissue sections were stained with hematoxylin and eosin (H&E) according to the standard procedure to detect the morphological changes in rats' brains.

### 2.6. ELISA

The levels of TNF-*α*, IL-6, IL-1*β*, and IL-18 in the brain tissue sample from each group were determined using ELISA according to the manufacturer's protocol (R&D Systems) at room temperature.

### 2.7. Brain-Water Content

After MCAO, the rats brains were quickly placed on ice, and it was recorded as wet weight. Then the brains were incubated at 110°C for 24 hours and then reweighed for the dry weight. The electronic analytic balance was used to weigh the brain weight. The formula for assessing the brain water content is as follows: ((wet weight − dry weight)/(wet weight)) × 100.

### 2.8. Terminal Deoxynucleotidyl Transferase dUTP Nick End Labeling (TUNEL) Assay

The brain tissue from different treatment groups was sectioned at 30 *μ*m thickness, dewaxed, and blocked in 3% H_2_O_2_ for 5 min and finally stained with TUNEL kits. The apoptosis ratio of brain tissue was determined by TUNEL Assay Kits (R&D Systems) according to manufacturer's instruction. The results were averaging the number of apoptotic cells/field at ×400 magnification, and the neuron apoptosis was represented as apoptosis index calculated as follows: apoptosis index = the number of TUNEL − positive cells/the total number of cells.

### 2.9. Statistics

All results were analyzed by GraphPad 6 software (GraphPad Software) and expressed as mean ± SEM. Data statistical significance was determined by one-way analysis of variance (ANOVA), and *t*-tests were used to make a comparison. *p* < 0.05 was considered statistically significant.

## 3. Results

### 3.1. Downregulation of HMGA2 Ameliorated the Neuron Function and Brain Injury in Cerebral Infarction Rats

To functionally analyze the role of HMGA2 in cerebral infarction, the model of middle cerebral artery occlusion (MCAO) in rats was constructed. After cerebral infarction, the rats were transfected with two different lentiviruses carrying sh-NC and sh-HMGA2. The relative HMGA2 mRNA expression was determined by qPCR (Figure 1(a)). Densitometric analysis of the bands from the western blots shown an increased HMGA2 level after cerebral infarction and a decrease in HMGA2 expression in the MCAO + sh-HMGA2 group (Figure 1(b)). The water content in the damaged brain was used as a measure of edema after cerebral infarction. After cerebral infarction, the water content in the brain was remarkably higher than in the control group. Transfection with sh-HMGA2 resulted in obviously suppressed brain water content in the cerebral infarction condition (Figure 1(c)). In addition, the neurobehavioral function evaluation in NSS scores of the MCAO + sh-HMGA2 group was significant improved after brain injury compared to the scores of the MCAO group (Figure 1(d)). The TTC staining indicated that the brain infarct areas in the MCAO group was notably increased in comparison with the control group. sh-HMGA2 treatment evidently attenuated it (Figure 1(e)). At the hippocampus, the neuronal cells were disorderly arranged and became a pyknotic nucleus and vacuole around the nucleus, and the interstitial edema was obvious. In contrast, sh-HMGA2 treatment reduced the brain infarction induced neuronal morphology changes and ameliorated the interstitial edema (Figure 1(f)). There were no significant morphological changes in the control group. Together, these results demonstrated that inhibition of HMGA2 ameliorated the neuron function and brain injury in cerebral infarction rats.

### 3.2. The Inhibition of HMGA2 Attenuated the Inflammatory Response of Cerebral Tissue in Cerebral Infarction Rats

To further investigate the protective effects of HMGA2 downregulation on cerebral infarction, the expression levels of inflammatory cytokines in rat brain were quantified by qPCR and ELISA. As shown in Figures 2(a) and 2(b), the relative mRNA expression and protein expression of TNF-*α*, IL-6, IL-1*β*, and IL-18 were significantly promoted after brain injury, and downregulation of HMGA2 obviously suppressed the expressions of inflammatory cytokines. These results indicated that HMGA2 alleviated the damage associated with cerebral infarction-induced inflammatory response.

### 3.3. Downregulation of HMGA2 Suppressed the Level of Hippocampal Neuron Apoptosis in Cerebral Infarction Rats

To investigate the mechanism underlying the neuroprotective effect of HMGA2 on cerebral infarction, hippocampal neuron apoptosis was measured using TUNEL staining. After MCAO operation, brain injury induced DNA fragmentation and increased TUNEL-positive cells in the MCAO group compared with the control group. In contrast, the TUNEL-positive cell number was remarkably suppressed in the MCAO + sh-HMGA2 group (Figure 3(a)). The western blot analysis was performed to detect the apoptosis-related proteins, such as Bax, cleaved caspase-3, and Bcl-2. The results indicated that Bax and cleaved caspase-3 expression levels were enhanced in the MCAO group and markedly decreased in the sh-HMGA2 treatment group. Moreover, the expression level of Bcl-2 was significantly upregulated in the sh-HMGA2 treatment group after brain injury (Figure 3(b)). These results suggest that inhibition of HMGA2 ameliorated the cerebral infarction-induced hippocampal neuron apoptosis.

### 3.4. Reduction of HMGA2 Expression Inhibits the Activation of TLR4/NF-*κ*B Signaling Pathway in Cerebral Infarction Rats

To explore whether HMGA2 regulates TLR4/NF-*κ*B pathway in cerebral infarction, the TLR4/NF-*κ*B pathway-related proteins were determined using western blot analysis. The results indicated that the expression levels of TLR4, p65, p-p65, and p-I*κ*B in cerebral infarction rats were significantly increased compared with the control group, which were remarkably attenuated in the MCAO + sh-HMGA2 group (Figure 4). Furthermore, the I*κ*B expression was downregulated following the MCAO operation, but the sh-HMGA2 treatment reversed this effect (Figure 4). These results suggested that downregulation of HMGA2 had a protective effect on the brain from cerebral infarction through mediating the regulation of the TLR4/NF-*κ*B pathway.

## 4. Discussion

In neurology clinical practice, cerebral infarction is a common disease with high disability and fatality rates [14]. The incidence rates of cerebral infarction or cerebral ischemic stroke are gradually increasing with aging and cerebrovascular disease progression [15]. This disease is usually accompanied by varying degrees of ischemia and anoxia which can cause malacia or necrosis of brain cells [16]. In addition, patients with acute cerebral infarction generally have neurological functional deterioration or progressive aggravation even after curative and timely treatment [17]. The middle cerebral artery occlusion (MCAO) is a classical animal model for studying cerebral infractions [18], which has many aspects of advantages, including small wounds to animals, operating easily, high repeatability, and brain edema significantly, and produces cerebral injury [19]. Using this model, this study first demonstrated that inhibition of HMGA2 exerted a neuroprotective effect on cerebral infarction, by reducing the brain infarct areas and protecting the brain from infarction-induced neuronal morphology changes and interstitial edema. Meanwhile, the results also showed that suppressed HMGA2 could attenuate the neurological dysfunction of brain injury rats and also markedly reduced infarct volume in the TTC experiment.

Cerebral infarction-induced brain injury is associated with inflammatory responses, which play a critical role in neuron dysfunction and apoptosis in the brain regions, and the anti-inflammatory therapy might be significant in cerebral infarction [20]. Multiple lines of evidence in clinical studies indicated that acute and prolonged inflammatory responses play a critical role in brain injury, and the reduction of the release of the cytokines including IL-1*β*, TNF-*α*, IL-6, or IFN-*γ* was beneficial for the brain injury therapy [21, 22]. A previous study demonstrated that cerebral infarction triggers the TLR signaling activation-induced inflammatory responses, further leading to the expression of NF-*κ*B-mediated inflammatory cytokines, such as IL-1, IL-6, IL-8, and TNF-*α* [23]. HMGA2 is a member of the high-mobility group box family which expressed in the microglial nucleus and serves as proinflammatory mediator. Previous studies have showed that the expression level of HMGB2 was increased in the serum of myocardial infarction patients and has a positive correlation with myocardial infarction severity and cellular apoptosis [24]. The functions of HMGB2 are widely reported in cardiovascular disease, but less research has been done in cerebral infarction. The high expression level of HMGB2 was closely associated with principal adverse cardiac events, and in-stent restenosis, and it promoted neointimal hyperplasia with femoral artery injury [25, 26]. Accumulated studies have reported that activating vascular smooth muscle cells and macrophages triggers the production and release of HMGB2 [25]. Conversely, inhibition of HMGB2 in cells or blocking their release could attenuate the immune response. These research are consistent with our findings, which showed that downregulation of HMGA2 alleviated the damage associated with cerebral infarction-induced inflammatory response and brain cellular apoptosis. Moreover, in the neural stem or progenitor cells, HMGB2 highly affected the epigenetic landscape during the perinatal transition from cortical neurogenesis to gliogenesis [27]. Our results presented here suggested a role for HMGB2 in neuron cellular repair dynamics, suggesting a novel HMGB2-dependent effect in the cerebral.

HMGB2 has been implicated in numerous cellular processes such as cell survival, differentiation, DNA replication, recombination, repair, transcription, inflammation, migration, and cell signaling [28]. TLR4/NF-*κ*B signaling pathway was connected with cellular processes in neurons and activated secondary inflammation in strokes [29, 30]. TLR4 is involved in regulating inflammation through adaptor proteins to trigger NF-*κ*B signaling and activate antigen presentation and T cell immune responses [31, 32]. In TLR4 knockdown stroke animal models, the infarct sizes were significantly decreased. This study demonstrated that TLR4/NF-*κ*B pathway was highly activated in the cerebral infarction rats. In contrast, downregulation of HMGA2 effectively suppressed TLR4/NF-*κ*B pathway in the animal of cerebral injury.

## 5. Conclusion

In summary, the current study demonstrated that downregulation of HMGB2 decreased the infarct size, inflammatory responses, and apoptosis in cerebral injury and had neuroprotective effects against cerebral infarction-induced brain damage. Finally, these results indicated that downregulation of the TLR4/NF-*κ*B pathway after ischemia by HMGB2 inhibition was a potential mechanism for the neuroprotective effect of cerebral injury.

## Figures and Tables

**Figure 1:** The effects of HMGA2 on neuron function and brain injury in cerebral infarction rats. (a) Quantitative PCR was performed to examine the mRNA expression level of HMGA2. (b) Western blot was used to explore the protein expression level of HMGA2. (c) Cerebral tissue water content after cerebral infarction compared. (d) Neurological severity scores were evaluated the neuron function. (e) TTC staining was used to explore the infarct volumes after MCAO. (f) H&E staining to analysis the brain tissue sections in cerebral infarction rats. ^∗∗^*p* < 0.01 vs. sham or MCAO + sh-NC. ^∗^*p* < 0.05 vs. sham or MCAO + sh-NC. Data are expressed as mean ± SEM.

**Figure 2:** The effects of HMGA2 on brain injury induced inflammatory response. (a) Quantitative PCR was performed to examine the mRNA expression level of TNF-*α*, IL-6, IL-1*β*, and IL-18 cerebral infarction. (b) Western blot was used to explore the protein expression level of TNF-*α*, IL-6, IL-1*β*, and IL-18 after cerebral infarction. ^∗∗^*p* < 0.01 vs. sham or MCAO + sh-NC. Data are expressed as mean ± SEM.

**Figure 3:** The effects of HMGA2 on brain injury induced apoptosis. (a) Analysis of cellular apoptosis ratio on cerebral infarction rats that transfected with sh-HMGA2 or sh-NC. (b) Western blot was used to explore the protein expression level of apoptosis related protein after cerebral infarction. ^∗∗^*p* < 0.01 vs. sham or MCAO + sh-NC. Data are expressed as mean ± SEM.

**Figure 4:** The effects of HMGA2 on TLR4/NF-*κ*B signaling pathway activation in cerebral infarction rats. Western blot analysis of protein expression in the TLR4/NF-*κ*B signaling pathway after sh-HMGA2 or sh-NC transfection. ^∗∗^*p* < 0.01 vs. sham or MCAO + sh-NC. Data are expressed as mean ± SEM.

## Data Availability

All data generated or analyzed during this study are included in this published article.
